The article "Design and Manufacture of Data Gloves for Rehabilitation Training and Gesture Recognition Based on Flexible Sensors" was retracted in 2023. Reasons: signs of a paper mill; compromised peer review; unreliable results or conclusions.

# Design and Manufacture of Data Gloves for Rehabilitation Training and Gesture Recognition Based on Flexible Sensors

**DOI:** 10.1155/2021/6359403

**Published:** 2021-12-07

**Authors:** Kai Guo, Senhao Zhang, Shasha Zhao, Hongbo Yang

**Affiliations:** ^1^School of Biomedical Engineering (Suzhou), Division of Life Sciences and Medicine, University of Science and Technology of China, Hefei 230026, China; ^2^Suzhou Institute of Biomedical Engineering and Technology, Chinese Academy of Sciences, Suzhou 215163, China

## Abstract

This work takes the production and usage scenarios of the data glove as the research object and studies the method of applying the flexible sensor to the data glove. Many studies are also devoted to exploring the transplantation of flexible sensors to data gloves. However, this type of research still lacks the display of specific application scenarios such as gesture recognition or hand rehabilitation training. A small amount of experimental data and theoretical analysis are difficult to promote the development of flexible sensors and flexible data gloves design schemes. Therefore, this study uses the self-made flexible sensor of the research group as the core sensing unit to produce a flexible data glove to monitor the bending changes of the knuckles and then use it for simple gesture recognition and rehabilitation training.

## 1. Introduction

Gesture recognition technology mainly refers to the user's use of simple gestures to interact with the device. Gesture recognition devices can allow computers to understand human behaviour and intentions, thereby making people's lives more convenient. Gesture recognition technology has a wide range of applications in assisted driving, sign language cognition, machine control, and other fields [1, 2].

Currently, the appearance of various types of sensors makes wearable electronic devices more diverse. According to the form of contact between the sensor and the human body, there are three types of sensor devices used in wearable devices: direct contact, noncontact, and embedded [3].

Chen et al. compared different sensors and different data gloves [4]. They mainly compared bending and stretching sensors, IMU inertial sensors, and magnetic sensors. By comparison, it is found that the bending sensor and the stretching sensor have better deformability, and the flexibility characteristics have good adaptability to the palm, so they are very suitable for hand posture estimation. Although, IMU inertial sensors and magnetic sensors have a certain impact on wearing. Because of its high mechanical strength, data gloves using these two sensors have a longer service life.

The direct contact sensor touches the surface of the skin and detects physical signs through electrical signals or chemically analyzes human sweat. Noncontact sensors are usually placed in some common wearable clothing and accessories [5, 6] and are currently the main sensor type used in wearable devices. Embedded sensors will be implanted inside the human body to monitor the physiological information of human organs, joints, and other parts.

The article "Design and Manufacture of Data Gloves for Rehabilitation Training and Gesture Recognition Based on Flexible Sensors" was retracted in 2023. Reasons: signs of a paper mill; compromised peer review; unreliable results or conclusions.

Divided by the type of material properties, sensors can be divided into two categories: rigid sensors and flexible sensors.

Rigid sensors are usually based on hard materials such as resin and metal. When the rigid sensor is in contact with the epidermis, it will give people an obvious foreign body sensation and limit the free movement of the limb joints. Moreover, the poor fit also affects the accuracy of rigid sensor data.

Flexible sensors are a new type of sensors in recent years. They usually use fabrics and films as substrates, which have a good fit with human skin and can ensure a more comfortable wearing experience. The stability and durability of flexible sensors are constantly improving, and they have very broad application potential.

By analyzing the inherent characteristics and movement characteristics of a human finger, a flexible stretch sensor suitable for collecting finger bending can be designed. By collecting the resistance change caused by the sensor stretch, the bending state of each finger is obtained. Designing software and hardware and related appearances can complete the design and production of data gloves. By designing different algorithms, the static and dynamic motion states of the fingers can be collected. At the same time, the application of data gloves in rehabilitation training is discussed [7–10].

Most of the existing data gloves were used in VR and scene interaction [11, 12], and few of them use data gloves in gesture recognition [1–4]. This study focused on the research of gesture recognition and related applications based on flexible sensors. Through the design and processing of the flexible sensor, after testing the tensile and repeatability characteristics of the sensor, a flexible sensor suitable for fingers was completed. Through training, the gesture recognition of the data glove using the flexible sensor was completed. At the same time, some attempts have been made to apply data gloves to rehabilitation training.

## 2. Materials and Methods

The basis of gesture recognition is the hardware design of gesture recognition, which mainly includes the design of the data glove bending sensor, and the circuit design and production of the data acquisition module [13–17].

For the collection of finger bending, commonly used sensors include inertial-based acceleration sensors and flexible stretch and bend sensors. Considering the comfort of wearing, we use the flexible sensor we designed, combined with the design of the circuit and the appearance of the glove, so as to complete the manufacture of our data glove.

The article "Design and Manufacture of Data Gloves for Rehabilitation Training and Gesture Recognition Based on Flexible Sensors" was retracted in 2023. Reasons: signs of a paper mill; compromised peer review; unreliable results or conclusions.

### 2.1. Design and Test of Flexible Sensor

The bending sensor of the data glove is the basic equipment for collecting data. We mainly collect the voltage ADC data change caused by the resistance change of the collected bending sensor [11, 12, 17–19]. This study mainly uses a flexible bending sensor coated with graphene, a new material, as a data acquisition sensor. The design of the flexible graphene sensor is shown in Figure 1.

We transferred the graphene to the flexible PDMS base to complete the production of the sensor. The completed bending sensor is shown in Figure 2.

After the sensor is made, the actual performance of the sensor was tested through a tensile experiment. The experiment is shown in Figure 3. Before stretching, the sensor length was L1, after stretching the length reaches L2, and the stretching rate was equal to (L2-L1)/L1.

The stretching process is shown in Figure 4. We used a stretcher to stretch and use a multimeter to test the resistance change during the stretching process.

### 2.2. Data Acquisition and Transmission Hardware

The main output of the finger bending acquisition sensor is resistance, which needs to be converted into a voltage signal and amplified and filtered, and the resistance value is obtained after ADC collection. At the same time, the circuit uses CC2540s BLE chip as a processor to collect ADC electrical signals and transmit them via bluetooth [20–25]. The structure of the hardware is shown in Figure 5.

The signal processing uses two MCP6004 chips, which are 4-channel 1 MHz bandwidth low-power operational amplifiers. The sensor signal acquisition and amplifying circuit composition of the data glove is shown in Figure 6.

In order to adapt to the situation of wearing left and right hands, we reserve six interfaces in the circuit, and the hardware we designed is shown in Figure 7.

As shown in Figure 7, P5 and P6 correspond to the thumb sensors, and both P5 and P6 are used to connect sensor E, which can be adapted to the left and right hands, respectively. P1 to P4 connect the other four fingers.

The MCP6004 is a quad general purpose op-amp because we use six sensors; so in this article, we used two MCP6004 chips. We used an Analog Devices analog to digital converters chip called AD7927BRU to transmit the collected signals to the Bluetooth master chip through the SPI interface. The signal amplification and ADC acquisition circuit are shown in Figure 8.

The article "Design and Manufacture of Data Gloves for Rehabilitation Training and Gesture Recognition Based on Flexible Sensors" was retracted in 2023. Reasons: signs of a paper mill; compromised peer review; unreliable results or conclusions.

The circuit board we made is shown in Figure 9. In the interface, e and f are connected; corresponding to the thumb, when wearing the left or right hand, only connect the sensor to E1 or E2, respectively. The remaining four ports correspond to the remaining four fingers.

As shown in the hardware physical drawing of the data glove, the size of the hardware part of the data glove is 34 mm^*∗*^25 mm. Coupled with a 150 mAh lithium battery, the overall thickness is about 5.5 mm, which can be placed on the palm of the hand without affecting the movement of the fingers. The hardware is written with BLE combined with low-power software, which produces less heat. The design of the data glove considers the convenience of wearing, and the hardware is placed in the palm of the hand.

### 2.3. Design and Testing of Data Gloves

Considering wearability and breathability, the glove body is designed as shown in Figure 10. The bending sensor of each finger is placed in the cloth interlayer on the back of the hand. The sensor is connected to the hardware through wires and interfaces. The gloves on the inner side of the finger joints are hollowed out to ensure the breathability and sports comfort of the gloves.

### 2.4. Gesture Recognition Using Flexible Sensor Gloves

For gesture recognition based on sensor data, commonly used data processing methods include template matching methods and neural network algorithms. As shown in Figure 11, we select 1–10 gestures commonly used by Chinese people for data collection and gesture recognition algorithm processing.

In model training session, we collected a training set containing 20,000 data samples from two volunteers, both of them repeatedly worn the glove 50 times and each of all the 10.

Gestures will be continuously performed 20 repetitions during every time wearing (2 volunteers × 50 times wearing × 10 gestures × 20 repetitions = 20,000 data samples).

#### 2.4.1. Template Matching Gesture Recognition

Template matching is a very common identification method. This method was originally used for image processing. The process of this algorithm is to search for small targets in a large image, and the benchmark for finding small targets is the degree of matching with the template [1–3].

Template matching recognition is simple, and the principle is easy to understand, so it has become the most basic gesture recognition method. The principle of template matching is to use the bending data of the finger collected by the device to match the data with the calculated template and to identify it by measuring the similarity [8, 9].

The main implementation process of template matching is the process of finding the target image. The process is shown in Figure 12. Template matching can find the target according to the following steps [1, 8].

The article "Design and Manufacture of Data Gloves for Rehabilitation Training and Gesture Recognition Based on Flexible Sensors" was retracted in 2023. Reasons: signs of a paper mill; compromised peer review; unreliable results or conclusions.

First, the starting position of template *w* is at the upper left corner of image f, and the center of template *w* can be anywhere, but if it is on the four edges of image f, f needs to be filled, just like the dotted line in the figure. But, it is required that the filling width cannot exceed half of the template.

Then, the template *w* moves from the upper left corner to the lower right corner. Each time it moves one unit distance, the similarity between *w* and f can be obtained by calculation. The calculated similarity measure value should be saved in the result image. Then, you can see the matching value in every position in the result.

Finally, it is necessary to determine the processing and analysis process of the result image according to the matching algorithm used and then find the matching position to determine the position of the target image.

#### 2.4.2. Neural Network Gesture Recognition

The commonly used three-layer structure neural network is shown in Figure 13. It is a multilayer, forward recursive network model. It mainly includes the input layer, hidden layer, and output layer [10, 13, 14].

There are 10 types of recognized gestures, so the output layer has 10 neurons. The activation function selects the Softmax function commonly used in multiclassification problems. The number of neurons in the hidden layer can be roughly determined by some strategies, and a better value can be finally selected through constant adjustment [1, 10].

We refer to the following formula to get a rough estimate:

(1) $$\begin{array}{c} n_{\text{hidden}}=\sqrt{n_{\text{input}}\times n_{\text{ouput}}}+m. \end{array}$$

In the formula, *n* was the number of neurons in the network layer shown by its subscript, and *m* is an integer in the range (0, 10). We set the number of neurons in the hidden layer to 12. We used cross-entropy loss as the loss function [14, 15].

We used 90% of the training set data for training and the remaining 10% for the verification set and used a 5-fold cross-validation method to test and adjust the structure of the neural network. The input layer contained 20 neurons, and the hidden layer contains 12 neurons. Take the ReLU function as the activation function. The output layer contains 10 neurons, with Softmax function as the activation function [1, 16]. Part of the parameter settings of the model: the loss function is the cross-entropy loss, the “Adam” optimization method is selected, the batch size is selected as 5, and the epoch is selected as 200 times. We choose the cross-entropy loss function and the “Adam” optimization method. The batch size was selected as 5, and the epoch was selected as 100 times.

The article "Design and Manufacture of Data Gloves for Rehabilitation Training and Gesture Recognition Based on Flexible Sensors" was retracted in 2023. Reasons: signs of a paper mill; compromised peer review; unreliable results or conclusions.

## 3. Results and Discussion

### 3.1. Stretch Test of Flexible Sensor

Test the parameters of the manufactured flexible sensor. Test each of the five sensors to be used and record the resistance values at different stretch rates. The resistance change with the stretch rate is shown in Figure 14.

The results and discussion may be presented separately or in one combined section and may optionally be divided into headed subsections.

### 3.2. Sensor Bending and Repeatability Test

After the glove body is made, Bluetooth data are collected through the mobile app to realize the monitoring of finger curvature data. To test the collection of the bending of a single finger, the index finger moved to 0°, 45°, 90°, and 135° respectively, as shown in Figure 15 for different finger movement states.

According to the different bending states of the index finger, the amplified electrical signals are collected, as shown in Figure 16.

For the index finger sensor under different bending states, three repeated experiments were carried out, and the signal values of 0°, 45°, 90°, and 120° were collected. The results of the repeated collection of three bending experiments are shown in Figure 17.

For gloves with flexible sensors, experiments have found that the sensors have good repeatability and can be used to judge different finger movement states.

### 3.3. Gesture Recognition Algorithm and Accuracy

After the template matching model is built, we match the samples of the test set with the trained various gesture templates and obtain the predicted gesture category according to the above method. The test results are given in Table 1.

From the results, the overall recognition accuracy rate reached 95.7%. For gestures with obvious features such as “1,” “5,” and “10,” the gesture shape is relatively stable, and the recognition accuracy will be higher.

The samples are tested in the trained neural network, and the recognition results of the same data are given in Table 2.

From the results, the overall recognition accuracy rate is over 98%. This shows that the flexible sensor can monitor static gesture features well and has good stability.

### 3.4. New Mirror Rehabilitation Training

In addition to being used for gesture recognition, data gloves can also be used for mirror rehabilitation training. The two-way flexible rehabilitation training glove device used is shown in Figure 18.

One of the commonly used rehabilitation training for hand function is called mirror training. Traditional mirror training is to use a mirror to let the patient see the movement of the uninhibited hand. In the mirror, it seems that the hand on the affected side is also moving to promote recovery. Use the above sports training gloves combined with data gloves to realize the healthy side hand driving the affected side hand and realize a new type of mirror training.

The article "Design and Manufacture of Data Gloves for Rehabilitation Training and Gesture Recognition Based on Flexible Sensors" was retracted in 2023. Reasons: signs of a paper mill; compromised peer review; unreliable results or conclusions.

Compile the host computer software and write the Bluetooth protocol communication to realize the use of flexible data gloves to control the rehabilitation training gloves. Realize palm-opening, fist-making, and finger-to-finger training are shown in Figure 19.

After the test, shown in Figure 19, it is verified that the data glove based on the flexible sensor can be well applied in the hand function rehabilitation training.

## 4. Conclusions

This study designs a data glove using a flexible bending sensor and completes gesture recognition and preliminary use in rehabilitation training.

First, a flexible bending sensor that can be used to monitor the bending state of the finger is designed. The performance of the sensor is verified through experiments, and the acquisition hardware using BLE communication is designed to acquire the bending state of the finger in real time. Using the bending sensor and the designed hardware, the production of the data glove is completed. By collecting different bending state data of a single finger, it is verified that the flexible bending sensor is suitable for the collection of finger bending data.

Then, by collecting a large amount of data, an algorithm based on template matching and a gesture recognition algorithm based on the neural network are built. The judgment accuracy of gestures through experiments meets general needs.

Finally, we use the communication protocol to combine data gloves and sports rehabilitation gloves to achieve a new type of hand mirror training mode.

## Figures and Tables

**Figure 1:** Design of the flexible stretch resistive sensor [3, 4].

**Figure 2:** Flexible sensors for data gloves.

**Figure 3:** Schematic diagram of sensor stretching.

**Figure 4:** Tensile experiment of the sensor.

**Figure 5:** The main components of the acquisition hardware.

**Figure 6:** Data acquisition and amplifying circuit composition.

**Figure 7:** Schematic diagram and circuit diagram of the data glove.

**Figure 8:** Signal amplification and ADC acquisition circuit.

**Figure 9:** The circuit part of the data glove.

**Figure 10:** The main components of the data glove.

**Figure 11:** Hand position from 1 to 10.

**Figure 12:** The mechanism of template matching [1, 8].

**Figure 13:** The three-layer structure neural network [1, 10, 14].

**Figure 14:** Resistance change under different stretch rates.

The article "Design and Manufacture of Data Gloves for Rehabilitation Training and Gesture Recognition Based on Flexible Sensors" was retracted in 2023. Reasons: signs of a paper mill; compromised peer review; unreliable results or conclusions.

**Figure 15:** Different bending state of the index finger.

**Figure 16:** Signal amplitude of different bending states.

**Figure 17:** Signal amplitude of different bending states in three tests.

**Figure 18:** Two-way movement rehabilitation gloves.

**Figure 19:** Mirror training using flexible sensor gloves. (a) Hand open. (b) Hand close. (c) Index finger to finger. (d) Middle finger to finger. (e) Ring finger to finger. (f) Pinky finger to finger.

**Table 1:** Accuracy of static gesture recognition using template matching.

	1	2	3	4	5	6	7	8	9	10	Accuracy (%)
1	299	1	0	0	0	0	0	0	0	0	99.7
2	4	291	5	0	0	0	0	0	0	0	97.0
3	0	5	287	6	2	0	0	0	0	0	95.7
4	0	0	0	292	5	3	0	0	0	0	97.3
5	0	0	0	0	300	0	0	0	0	0	100.0
6	0	0	0	0	2	292	4	2	0	0	97.3
7	0	0	0	4	2	0	292	2	0	0	97.3
8	0	0	0	0	0	0	4	296	0	0	98.7
9	0	0	1	0	0	0	2	4	292	2	97.3
10	0	0	0	0	1	0	0	0	0	299	99.7

**Table 2:** Accuracy of static gesture recognition using neural networks.

	1	2	3	4	5	6	7	8	9	10	Accuracy (%)
1	300	0	0	0	0	0	0	0	0	0	100.0
2	1	298	1	0	0	0	0	0	0	0	99.3
3	0	2	298	0	0	0	0	0	0	0	99.3
4	0	0	0	296	3	1	0	0	0	0	98.7
5	0	0	0	0	299	1	0	0	0	0	99.7
6	0	0	0	0	0	298	1	1	0	0	99.3
7	0	0	0	0	0	0	298	2	0	0	99.3
8	0	0	0	0	0	0	1	299	0	0	99.7
9	0	0	1	0	0	0	0	0	299	0	99.7
10	0	0	0	0	0	0	0	0	0	300	100.0

## Data Availability

The data used to support the findings of this study are available from the corresponding author upon request.
